# Potential Fault Diagnosis Method and Classification Accuracy Detection of IGBT Device Based on Improved Single Hidden Layer Feedforward Neural Network

**DOI:** 10.1155/2021/6036118

**Published:** 2021-09-30

**Authors:** Jie Wu, Xiaojuan Chen, Zhaohua Zhang

**Affiliations:** ^1^College of Electronic Information Engineering, Changchun University of Science and Technology, Changchun 130022, China; ^2^Beihua University, School of Electrical and Information Engineering, Jilin 132021, China

## Abstract

Insulated Gate Bipolar Transistor (IGBT) is a high-power switch in the field of power electronics. Its reliability is closely related to system stability. Once failure occurs, it may cause irreparable loss. Therefore, potential fault diagnosis methods of IGBT devices are studied in this paper, and their classification accuracy is tested. Due to the shortcomings of incomplete data application in the traditional method of characterizing the device state based on point frequency parameters, a fault diagnosis method based on full frequency threshold screening was proposed in this paper, and its classification accuracy was detected by the Extreme Learning Machine (ELM) algorithm. The randomly generated input layer weight *ω* and hidden layer deviation lead to the change of output layer weight *β* and then affect the overall output result. In view of the errors and instability caused by this randomness, an improved Finite Impulse Response Filter ELM (FIR-ELM) training algorithm is proposed. The filtering technique is used to initialize the input weights of the Single Hidden Layer Feedforward Neural Network (SLFN). The hidden layer of SLFN is used as the preprocessor to achieve the minimum output error. To reduce the structural risk and empirical risk of SLFN, the simulation results of 300 groups of spectral data show that the improved FIR-ELM algorithm significantly improves the training accuracy and has good robustness compared with the traditional extreme learning machine algorithm.

## 1. Introduction

Insulated Gate Bipolar Transistor (IGBT) is a power semiconductor device consisting of BJT and MOS, which has been fully applied to high-precision fields, such as new energy power generation, wind power, electric locomotive traction, and electric vehicles [1, 2]. In these applications, IGBT devices typically work in a harsh operating environment. It is closely related to system stability. However, such semiconductor devices inevitably produce potential defective devices in mass production, this part of the device has a short life, and there is a major hidden danger for the stability of the system. Failure may result in irreparable losses. So, facing severe reliability challenges, its reliability assessment is increasingly focusing on academia and industrial community [3–5]. Therefore, the fault diagnosis method of IGBT devices is studied, maintaining overall system stability, reducing economic losses and casualties related to employees, and is significant.

The original fault diagnosis method is primarily diagnosed with the hard fault of the short-circuit open circuit in the actual circuit [6]. It is not possible to improve the defects inside the device in good reactive devices. The device is placed in an environment of the power cycle or a high and low temperature, and the obtained electrical parameter is still in line with the performance indicator of the device, but during the test, it has caused a damage to the device, and the standard of nonlossless diagnosis is not met. The potential fault diagnosis caused by internal defects has been raised in recent years. Some experts learned from the perspective of theoretical analysis to apply low-frequency noise applications on the potential fault diagnosis of electronic devices, but it is only limited to this. Judging basis for potential fault diagnosis, only a few universities at home and abroad have studied low-frequency noise, so there is currently a potential fault diagnosis of IGBT devices through low-frequency noise detection, and there is no accurate and agreed evaluation criteria at home and abroad. In addition to this difficulty, it is also necessary to consider the source of IGBT devices, manufacturers, product batch, and other factors. All of them may affect the experimental results and evaluation standards, which also adds a certain difficulty in potential fault diagnosis.

Since the problem of potential fault diagnosis of IGBT devices is particularly important. In recent years, the feedforward neural network of single hidden layers has attracted extensive attention in many engineering disciplines [7]. It is widely used in digital signal and image processing, complex system modeling, adaptive control, data classification, and information retrieval by appropriately selecting the number of nodes in the hidden layer and the output layer and training input and output weight. In practical applications, techniques for training SLFN weights are very important in order to ensure the good performance of SLFN. The most popular training technology for SLFN is based on the BP algorithm [8], which is easy to implement BP from the output layer of SLFN to the hidden layer. However, slow convergence limits the application of BP in function approximation, pattern recognition, classification, and data compression. In addition, the sensitivity of SLFNs using BP training to input interference and data is another important issue. In 2004, Professor Huang Guangbin proposed a limit learning machine (ELM) algorithm [9], randomly allocated SLFN input weight and hidden layer deviation and the overall deemed linear network, and then calculated the output weight of SLFN by using the generalized inverse matrix of the hidden layer output matrix. However, in contrast, ELM has extremely fast learning speed in many cases and has good performance. However, by observation, the SLFN robustness of ELM training is poor because SLFN signals to signal the data containing noise; due to the influence of input interference, the change of the hidden layer output matrix is sometimes very large, which will also cause SLFN output rights. The value matrix change is large. Therefore, in this article, we propose a new FIR-ELM algorithm that uses filtering techniques when initializing the input homogenesis and improves SLFN's stability, balance, and reduced structural risks and experience risks of noise data processing, thereby enhanced nonlinear neural networks are important to improving the detection accuracy of improving fault diagnosis in input disturbances.

In summary, the research content of this article is shown in Figure 1.

## 2. Fault Diagnosis Method Based on Full Frequency Band Threshold Screening

The use of some point frequency parameter expressions to obtain the size of the results, as a criterion for screening good and bad, is currently a method of characterizing the reliability of low-frequency noise. For example, calculate *V*_*n*_ (the noise power spectrum value at 1 Hz), *γ*=(*V*_*n*(10)_/*V*_*n*(1)_) (the ratio of the noise power spectrum at 10 Hz to 1 Hz), and so on. However, this method ignores the particularities and differences between different devices, and the 1/*f* noise in different devices will have different manifestations, resulting in different exponential coefficient gamma in the 1/*f* noise parameter. In this case, only low-frequency noise near a single frequency of 10 Hz can be detected, and low-frequency noise at other frequencies cannot be detected. Therefore, this screening evaluation standard is not yet complete and comprehensive, and the detection sensitivity is insufficient. Based on the disadvantages of this method, this article expands the scope to the noise power spectrum of the full frequency band of the IGBT device and calculates its effective value to characterize the performance of the IGBT device and realize the diagnosis of potential faults.

Based on the three-level inverter, IGBT has a lower reverse blocking voltage, and its internal silicon chip has lower switching loss and forward voltage drop, so this article mainly focuses on the IGBT devices in the three-level inverter. For fault diagnosis, the inverter contains 12 IGBT components, see Figure 2. Each phase will switch between three levels (+Vdc/2, 0, −Vdc/). In this structure, these IGBTs are connected to the neutral point (MP) through two clamping diodes, so the maximum voltage on the IGBT is limited to half of the maximum DC link voltage (Vdc/2).

During the experiment, 300 IGBT devices of the same manufacturer, batch, and production process were selected for full-band noise testing. Take the average of the spectral values corresponding to each frequency to form a set, calculate the mean square error *σ*_*i*_ of the set, and plot the result as a line to show the spectrum value of the entire frequency band, as shown in the solid line in Figure 3.

In order to obtain the diagnostic criteria for potential faults, a range of upper and lower limits is required [10, 11], and the calculation formula for a single-frequency point is as follows:

(1) $$\begin{array}{c} {\bar{S}}_{N}=\sum_{i=1}^{N}\frac{S_{i}}{N}, \end{array}$$

(2) $$\begin{array}{c} {\bar{S}}_{Nu}={\bar{S}}_{N}+\alpha \sigma , \end{array}$$

(3) $$\begin{array}{c} {\bar{S}}_{Nd}={\bar{S}}_{N}-\beta \sigma . \end{array}$$

Equation (1) is the abovementioned calculation formula for averaging the spectrum value of the frequency point, where the number of inverters is *N*; here, it refers to 300 in the experiment; then, calculate the spectrum band by equation (2). The spectrum value corresponds to the frequency point in the upper limit of the range. *α* mentioned in the formula is a dynamic coefficient, which represents the upper threshold of the spectrum band. Adjusting the value of *α* can change the range of the upper limit of the spectrum. In the same way, use formula (3) to calculate the spectrum value corresponding to the frequency point in the lower limit of the spectral band range, and then, adjust the range of the lower limit of the spectral band through the lower limit threshold *β*.

The final calculated result is shown in Figure 3. The range between the dashed line and the thick dotted line in the figure is the full frequency band range of the inverter.

### 2.1. Determination of the Screening Thresholds *α* and *β*

Assuming that, under this condition (that is, *n* is the total capacity of the sample, *c* is the confidence level, and *p* is the pass probability), the method of calculating the upper and lower thresholds *α* and *β* of low-frequency noise is as follows:

Based on the related mathematical theory in probability [12], it can be assumed that there is a sample *x*(*x*_1_, *x*_2_,…, *x*_*n*_), which is composed of *n* electronic components, and a regional range *G*(*x*_1_, *x*_2_,…, *x*_*n*_) is defined according to the sample, and solve the noise amplitude represented by *P*([*x*_1_, *x*_2_,…, *x*_*n*_]) to make it greater than or equal to the given upper limit probability.

For the normal distribution *N*(*μ*, *σ*^2^) with unknown mean and variance, the unbiased estimation method can be used to calculate it:

(4) $$\begin{array}{c} \bar{x}=\frac{1}{n}\sum_{i=1}^{n}x_{i}, \end{array}$$

(5) $$\begin{array}{c} {\left(S^{*}\right)}^{2}=\frac{1}{n}\sum_{i=1}^{n}{\left(x_{i}-\bar{x}\right)}^{2}, \end{array}$$

where *S*^*∗*^ represents the degree of dispersion of sample elements and $\bar{x}$ represents the average value of sample elements, and equation (6) can represent that, in *n* samples, the low-frequency noise index is not less than $\bar{x}+\alpha S^{*}$:

(6) $$\begin{array}{c} \frac{1}{\sqrt{2\pi \sigma }}\int_{-\infty }^{\bar{x}+\alpha S^{*}}e^{-\left({\left(x-\mu \right)}^{2}/2\sigma^{2}\right)}\text{d}x=\frac{1}{\sqrt{2\pi }}\int_{-\infty }^{\bar{x}-\mu +\alpha S^{*}}e^{-\left(t^{2}/2\right)}\text{d}t, \end{array}$$

(7) $$\begin{array}{c} \frac{1}{\sqrt{2\pi }}\int_{-\infty }^{\mu_{p}}e^{-\left(t^{2}/2\right)}\text{d}t=p, \end{array}$$

(8) $$\begin{array}{c} \bar{x}-\mu +\alpha S^{*}\geq \mu_{P}, \end{array}$$

(9) $$\begin{array}{c} \frac{-\left(\left(\bar{x}-\mu \right)/\left(\sigma /\sqrt{n}\right)\right)+\mu_{p}\sqrt{n}/\sigma }{\sqrt{\left(\left({\left(\left(n-1\right)/S^{*}\right)}^{2}\right)/\sigma^{2}\right)/\left(n-1\right)}}\leq \alpha \sqrt{n}, \end{array}$$

(10) $$\begin{array}{c} \alpha \sqrt{n}=t_{\left(n-1,\mu_{p}\sqrt{n}\right)c}. \end{array}$$

In order to satisfy formula (7), look for a specific value of *μ*_*p*_ in the *N*(0,1) distribution function table. The low-frequency noise in *n* samples constitutes a total set. Equation (8) represents the result that the index value is not less than $\bar{x}+\alpha S^{*}$ and the ratio is not less than *p*. After conversion, equation (9) is obtained. Observation shows that the equation obeys the distribution of $t_{\left(n-1,\mu_{p}\sqrt{n}\right)}$. Checking the table shows that when $\alpha =t_{\left(n-1,\mu_{p}\sqrt{n}\right)c}$, it satisfies $P\left(t<t_{\left(n-1,\mu_{p}\sqrt{n}\right)}\right)=c$, that is, formula (10) is obtained, and after simplification, solution expression (11) of the final upper threshold is obtained:

(11) $$\begin{array}{c} \alpha =\left(t_{\left(n-1,\mu_{p}\sqrt{n}\right)}/\sqrt{n}\right). \end{array}$$

### 2.2. Full Band Threshold Screening Standard

Based on the frequency band range shown in Figure 3, the potential faults of the inverter can be divided into the following three categories:

  If$\;S\leq {\bar{S}}_{N\;d}$, the inverter is a Class I device
  If ${\bar{S}}_{N\;d}<S\leq {\bar{S}}_{N\mu }$, the inverter is a Class II device
  If $S>{\bar{S}}_{N\mu }$, the inverter is a Class III device

The noise power spectral density of Class I devices is less than the lower limit of the threshold, indicating that the noise value is very small and reflecting the least surface and internal defects and the best performance; the noise power spectrum density of Class III devices is greater than the calculated upper threshold of the threshold, indicating the noise value. It is very large and contains many types of noise, and its performance is poor. Although it can be used, it has a short service life and is easily damaged.

## 3. Fault Classification Accuracy Detection Based on Extreme Learning Machine

### 3.1. Extreme Learning Machine

Traditional classification algorithms, such as *k*-nearest neighbor classification (KNN) algorithm and support vector machine (SVM) algorithm, each have their own strengths. The KNN algorithm uses all training sample points when predicting, and it is a nonsparse model. When the training set and test set are large, the efficiency is worrying. Although the SVM algorithm can solve machine learning problems in the case of small samples and improve generalization performance, it is sensitive to missing data and has no general solution to nonlinear problems. Therefore, in order to solve the above problems, an artificial neural network algorithm is proposed because it has strong robustness and fault tolerance to noise nerves, can fully approximate complex nonlinear relationships, and has strong parallel distributed processing capabilities, so it can deal with situations that contain a lot of parameters, but there may also be problems such as too long learning time or even failure to achieve the learning purpose. Based on these problems, this paper adopts a new and improved neural network algorithm to optimize learning time and improve learning efficiency.

Extreme Learning Machine (ELM): this algorithm was proposed by Professor Huang Guangbin of Nanyang Technological University and others in 2004. It is a machine learning method based on a single hidden layer feedforward neural network (SLFN) [13], but it is different from SLFN. It is a new and improved algorithm.

Figure 4 shows the structure of a single hidden layer feedforward neural network. The extreme learning machine abandons the shortcomings of the traditional feedforward neural network, that is, abandons the gradient algorithm to iteratively adjust the network parameters. The input layer weight and hidden layer deviation are randomly selected and then calculated by the Moore–Penrose (MP) generalized inverse matrix theory to obtain the output layer weight. Compared with the single hidden layer feedforward neural network, this random generation method reduces the training parameters, improves the learning speed, and strengthens the generalization ability. It has many advantages [14–18].

The traditional extreme learning machine algorithm has a single hidden layer and is usually compared with the support vector machine (SVM). Through comparison, it can be concluded that the extreme learning machine has the following characteristics:

(1) The parameter constraint conditions are simpler. Especially, when faced with the solution of nonlinear programming problems, the optimal hyperplane constructed by SVM usually does not pass through the origin of the feature space, and the following two constraints need to be met, such as the following equation:
  (12) $$\begin{array}{c} \left\{\begin{array}{c} \sum_{i=1}^{N}a_{i}y_{i}=0\\ 0\leq a_{i}\leq C,\;i=1,\ldots ,N \end{array}\right.. \end{array}$$
But when using the extreme learning machine for classification, only one condition needs to be met, that is, 0 ≤ *a*_*i*_ ≤ *C*,  *i*=1,…, *N*.
(2) Although the properties of the two algorithms are the same, both belong to the SLFN model, but ELM uses explicit mapping for feature characterization, while SVM uses implicit mapping. This process is relatively cumbersome for support vector machines.
(3) Through experimental analysis, it is proposed that the support vector machine optimization finds only suboptimal solutions. It only regards the boundary of maximizing classification as a category of single hidden layer network generalization ability. It is a special case, and it will not be in the end. No optimal solution was found.

For *N* arbitrary samples (*X*_*i*_, *t*_*i*_), *X*_*i*_=[*x*_*i*1_, *x*_*i*2_,…,*x*_in_]^*T*^ ∈ *R*^*n*^ and *t*_*i*_=[*t*_*i*1_, *t*_*i*2_,…,*t*_in_]^*T*^ ∈ *R*^*m*^, the mathematical model of the extreme learning machine with *L* hidden nodes can be expressed as

(13) $$\begin{array}{c} \sum_{i=1}^{L}\beta_{i}g\left(W_{i}\cdot X_{i}+b_{i}\right)=o_{j},\;j=1,\ldots ,N. \end{array}$$

In the formula, *W*_*i*_=[*w*_*i*1_, *w*_*i*2_,…,*w*_*in*_]^*T*^ is the input weight, *b*_*i*_ is the offset of the *i*^th^ hidden unit, *β*_*i*_ is the weight of the output, *N* is the sample size of the training set, *o*_*j*_ is the output classification result, and *g*(*x*) is the activation function.

In the ELM algorithm, the hidden layer can usually choose the following activation functions, as shown in Table 1:

In order to make the classification result *o*_*j*_ consistent with the real result *t*_*j*_, it can be expressed as

(14) $$\begin{array}{c} \sum_{j=1}^{N}\left\|o_{j}-t_{j}\right\|=0, \end{array}$$

that is, there are *β*_*i*_, *w*_*i*_,  and *b*_*i*_ so that

(15) $$\begin{array}{c} \sum_{i=1}^{L}\beta_{i}g\left(w_{i}\cdot X_{j}+b_{i}\right)=t_{j},\;j=1,\ldots ,N. \end{array}$$

The matrix is expressed as

(16) $$\begin{array}{c} H\beta =T. \end{array}$$

In the above formula, *H* represents the output of the hidden layer neuron, *β* represents the weight of the output, and *T* represents the expected output:

(17) $$\begin{array}{c} H\left(W_{L},b_{L},X_{L}\right)={\left[\begin{array}{c} \vdots \\ g\left(W_{L}\cdot X_{N}+b_{L}\right) \end{array}\right]}_{N\times L}, \end{array}$$

(18) $$\begin{array}{c} \beta ={\left[\begin{array}{c} \vdots \\ \beta_{L}{}^{T} \end{array}\right]}_{L\times m}, \end{array}$$

In order to get $\overset{\wedge }{w_{i}},\overset{\wedge }{b_{i}},\text{ and }\overset{\wedge }{\beta_{i}}$, make

(19) $$\begin{array}{c} \left\|H\left(\overset{\wedge }{W_{i}},\overset{\wedge }{b_{i}}\right)\overset{\wedge }{\beta_{i}-T}\right\|=\underset{W,b,\beta }{\text{min}}\left\|H\left(W_{i},b_{i}\right)\beta_{i}-T\right\|, \end{array}$$

where *i*=1,…, *L*, and the minimized loss function is

(20) $$\begin{array}{c} E=\sum_{j=1}^{N}{\left(\sum_{i=1}^{L}\beta_{i}g\left(W_{i}\cdot X_{j}+b_{i}\right)-t_{j}\right)}^{2}, \end{array}$$

where *H*[*N* × *L*] is a known matrix, and the output weight is unknown. Through ELM training and learning, the output weight matrix *β* is solved, and the least squares equation theory is used to get

(21) $$\begin{array}{c} \left\|H\hat{\beta }-T\right\|=\text{min}\left\|H\beta -T\right\|. \end{array}$$

Solve the following equation:

(22) $$\begin{array}{c} \hat{\beta }=H^{+}T. \end{array}$$

Combined with the singular value decomposition method [19], when *HH*^*T*^ is not singular,  *H*^+^=*H*^*T*^(*HH*^*T*^)^−1^.

In order to eliminate the error, the regularization coefficient *λ* is introduced, and the output weight is

(23) $$\begin{array}{c} \hat{\beta }=H^{T}{\left(HH^{T}+\lambda I\right)}^{-1}T. \end{array}$$

Finally, the output function of ELM is described as

(24) $$\begin{array}{c} y\left(x\right)=h\left(x\right)\hat{\beta }. \end{array}$$

To sum up, the extreme learning machine is different from the traditional neural network. The training problem of the original algorithm parameters is transformed into the calculation through the Moore–Penrose (MP) generalized inverse matrix theory, the linear equations are solved, and the least squares are obtained. The solution, which is the weight of the output layer in the algorithm, does not require repeated iterations during the training process, which saves learning and training time and improves generalization performance.

### 3.2. Experimental Results and Analysis

In order to verify the performance of the ELM algorithm for fault classification accuracy detection, this paper chooses to conduct experiments on the MatlabR2017a platform. According to the full-band threshold diagnosis and screening method introduced above, IGBT devices are divided into three categories: I, II, and III. Class I devices reflect the least surface and internal defects and have the most excellent performance; Class III devices have large noise values, contain many types of noise, and have poor performance.

For the three categories of IGBT devices, 100 devices are selected for each state for noise power spectrum detection, and 300 sets of spectrum data can be obtained, and 70% of the three categories of I, II, and III data are selected as training samples; the remaining 30% as the test sample, and the number of nodes in the ELM hidden layer is 3, and the sigmoid function is used as the activation function of the ELM hidden layer. The classification results are shown in Figure 5.

The actual test set classification is represented by the blue circle in the figure, and the predicted test set classification is represented by a red asterisk. If the two symbols are stacked together, it means that the algorithm predicts the classification result correctly. If the two symbols do not overlap, it means that the predicted classification in the actual situation is different, and the classification fails. From Figures 5(a)–5(c), it can be seen that, in this test set, the classification accuracy of the ELM model is 86.67%.

## 4. Accuracy Detection of Latent Fault Diagnosis Method Based on FIR-ELM

### 4.1. FIR-ELM Design Principle

The previous section proposed a learning algorithm for SLFN, called the extreme learning machine (ELM), in which the input weights and hidden layer deviation of SLFN are randomly assigned, and then, it is simplified into a linear network; using implicit, the generalized inverse of the layered output matrix calculates its output weight. It can be seen that ELM has a fast learning speed and produces good performance in many cases. However, SLFN trained with ELM has poor robustness when dealing with noisy data. For example, when input weights and hidden layer deviations are randomly assigned to an SLFN, sometimes due to the influence of input disturbances, the output matrix of the hidden layer changes greatly, which also causes the SLFN output weight matrix to change greatly. Based on the above problems, we propose a new robust training algorithm, which adds a memory with linear nodes and input tap delay lines for signal preprocessing. Since the output of each linear hidden node in SLFN is the sum of weighted input data, each node can be regarded as an FIR filter [20, 21]. The hidden layer is designed as a set of low-pass filters, high-pass filters, band-pass filters, band-stop filters, or other filter types which are used to process input data with interference and undesired frequency components. The preprocessing function of the hidden layer cannot only eliminate input interference and undesired frequency components. From the perspective of SLFN output, the structure and experience risk of SLFN can also be greatly reduced. Based on this function, the single hidden layer feedforward neural network structure diagram is shown in Figure 6.

On the basis of Section 2, we add *D* flip-flops to the input sequence to play the role of delayed storage.

From equation (13), we can see that the output of the *i*^th^ hidden node is

(25) $$\begin{array}{c} o_{i}\left(k\right)=\sum_{j=1}^{L}\omega_{ij}x\left(k-j+1\right)={\vec{\omega }}_{i}^{T}\vec{x}\left(k\right). \end{array}$$

It can be seen that formula (25) has a typical FIR filter structure, where the input weight set {*ω*_*ij*_} can be regarded as a set of filter coefficients or filter impulse response coefficients, and the output *o*_*i*_(*k*) is the result of the convolution sum of the filter impulse response and the input time series. The length of the filter is equal to the number of input data of the neural network. According to the related theory of signal processing, if the elements of the input weight vector are selected to be positive and symmetrical, then *ω*_*i*,*j*_ > 0 and

(26) $$\begin{array}{c} \omega_{i,j}=\omega_{i,\left(n-j+1\right)},\left\{\begin{array}{cc} j=1,2,\ldots ,\left(n-1\right)/2, & \text{ odd }n\\ j=1,2,\ldots ,n/2, & \text{even }n \end{array}\right.. \end{array}$$

It can be seen that this is a nonrecursive linear phase FIR filter. Since there are no poles, the output of all hidden nodes is stable and can achieve a smaller accuracy error than other types of filters.

Below we consider how to design to enable each hidden node to perform the filtering function. Here we use MATLAB to develop a look-up table, which contains all possible SLFN input weight sets for low-pass filters, high-pass filters, band-pass filters, and other specified filters. According to our observation and understanding of the frequency spectrum of the input data, we know which frequency components should be deleted or retained, and then, we can select a set of appropriate parameters from the look-up table and assign them to the input weights of SLFN [22, 23].

If we want the *i*^th^ hidden node in SLFN as a low-pass filter, the expected frequency response is as follows:

(27) $$\begin{array}{c} H_{i\;d}\left(\omega \right)=\left\{\begin{array}{cc} 1e^{-j\omega \left(n-1\right)/2} & \left|\omega \right|\leq \omega_{c}\\ 0 & \omega_{c}<\left|\omega_{c}\right|<\pi \end{array}\right., \end{array}$$

where *ω*_*c*_ is the cutoff frequency of the low-pass filter to separate the low-frequency pass band and the high-frequency stop band. The impulse response of the truncated low-pass filter is

(28) $$\begin{array}{c} {\overset{⌢}{h}}_{i\;d}\left[k\right]=\frac{1}{2\pi }\int_{-\omega_{c}}^{\omega_{c}}e^{-j\omega \left(n-1\right)/2}e^{j\omega k}\text{d}w=\frac{\sin\left[\omega_{c}\left(k-\left(n-1\right)/2\right)\right]}{\pi \left(k-\left(n-1\right)/2\right)}, \end{array}$$

(29) $$\begin{array}{c} {\overset{⌢}{h}}_{i\;d}\left[k\right]={\overset{⌢}{h}}_{i\;d}\left[n-k+1\right]. \end{array}$$

Thus, the weight of the *i*^th^ hidden layer node *ω*_*ij*_ can be obtained as

(30) $$\begin{array}{c} \omega_{i1}={\overset{⌢}{h}}_{i\;d}\left[0\right],\omega_{i2}={\overset{⌢}{h}}_{i\;d}\left[1\right],\ldots ,\omega_{in}={\overset{⌢}{h}}_{i\;d}\left[n-1\right]. \end{array}$$

In summary, using such a hidden layer preprocessing program to filter out high-frequency interference can significantly reduce the SLFN structure and experience risks.

Based on the above discussion, we summarize the proposed FIR-ELM algorithm as follows:

  Step 1: assign input weights *ω*_*ij*_ according to formulas (28)–(30)
  Step 2: use (17) to calculate the hidden layer output matrix $\vec{H}$
  Step 3: calculate and output the weight matrix $\vec{\beta }$ according to (23)

### 4.2. Simulation Results

We also use the data in Section 3 to test the performance of the FIR-ELM algorithm. The results of the accuracy detection of the potential fault diagnosis method of the FIR-ELM algorithm based on the low-pass filter, high-pass filter and band-pass filter are as follows (see Figure 7).

In order to make the results more fair and reduce the influence of other factors, the data presented in the table are all the data obtained by averaging multiple experiments. From the comparison of the data of the three groups of dimensions in Table 2, it can be seen that, after adding the prefilter, compared with the original ELM algorithm, the diagnostic accuracy and running time have been significantly improved. Among them, the low-pass filter is used as the prefilter of the input weight for detection, which has the highest accuracy and the fastest running speed, which provides a more reliable classification standard for the potential fault diagnosis of IGBT devices.

## 5. Conclusion

This paper firstly studies the performance of IGBT devices in three-phase three-level inverters and proposes the use of full-band threshold screening methods as potential fault diagnosis criteria, which overcomes the shortcomings of incomplete data characterization and low classification sensitivity using point frequency parameters in the past. Then, through comparative analysis, a new type of the neural network algorithm of the extreme learning machine is proposed, and the basic theory of the extreme learning machine is introduced, using the method of the extreme learning machine to detect the accuracy of the potential fault diagnosis classification. Aiming at the problem that its robustness needs to be improved, a new training algorithm FIR-ELM is proposed. At this point, regard it as a kind of neural feedback network with linear nodes. Linear FIR filtering technology has been successfully used to design input weights. This makes the hidden layer of SLFN as the preprocessing of input data, which can effectively eliminate input interference, and undesirable signal components reduce output errors and reduce the experience risk and structural risk of SLFN. Simulation results show that the proposed FIR-ELM training algorithm has good robustness in noisy environments.

Later, we will further analyze the performance of IGBT devices in other inverters, study the types of faults in more situations such as two-level and three-level, and then better combine signal processing technology to diagnose faults and their diagnostic performance. Detection makes more precise judgments. At the same time, in view of the powerful functions of the ELM algorithm, we can design a suitable network structure according to the needs to solve many problems such as huge data and inefficiency.

## Figures and Tables

**Figure 1:** Block diagram of the presented research.

**Figure 2:** The research object of this paper. (a) Data acquisition device driver based on the USB bus. (b) Topological structure of the three-phase three-level inverter. (c) IGBT module material. (d) Internal diagram of the IGBT module.

**Figure 3:** Average spectrum of the full frequency band and spectrum range.

**Figure 4:** Single hidden layer feed forward neural network structure diagram.

**Figure 5:** The classification results of the test set based on ELM. (a) ELM-based test set classification total results. (b) ELM-based test set classification display. (c) Corresponding results of test set classification based on ELM.

**Figure 6:** Structure diagram of the single hidden layer feedforward neural network based on FIR-ELM.

**Figure 7:** FIR-ELM algorithm classification results' performance detection diagram. (a) Classification result of the FIR-ELM algorithm based on the preband stop filter. (b) Classification result of the FIR-ELM algorithm based on the preband-pass filter. (c) Classification result of the FIR-ELM algorithm based on the front high-pass filter. (d) Classification result of the FIR-ELM algorithm based on the front low-pass filter.

**Table 1:** Hidden layer activation function.

Name	Mathematical expression
Triangular	*g*(*ω*_*i*_, *b*_*i*_, *x*)=cos(*b*_*i*_ · *x*+*ω*_*i*_)
Gaussian	$g\left(\omega_{i},b_{i},x\right)=\sqrt{x-b_{i}+\omega_{i}{}^{2}}$
Radial basis	*g*(*ω*_*i*_, *b*_*i*_, *x*)=exp(−*ω*_*i*_ · *x* − *b*_*i*_)
Sigmoid	*g*(*ω*_*i*_, *b*_*i*_, *x*)=(1/(1+exp(*b*_*i*_ · *x*+*ω*_*i*_)))
Sine	*g*(*ω*_*i*_, *b*_*i*_, *x*)=((1 − exp(*b*_*i*_ · *x*+*ω*_*i*_))/(1+exp(*b*_*i*_ · *x*+*ω*_*i*_)))
Hardlim	$g\left(\omega_{i},b_{i},x\right)=\left\{\begin{array}{cc} 1， & b_{i}\cdot x\leq 0,\\ 0， & \text{others.} \end{array}\right.$

**Table 2:** Comparison of training accuracy, testing accuracy, and running time of different methods.

Classification	Training accuracy	Testing accuracy	Running time (s)
ELM	0.8857	0.8667	0.2166
FIR-ELM (band stop filter)	0.9205	0.9222	0.2003
FIR-ELM (band pass filter)	0.9422	0.9444	0.2001
FIR-ELM (high-pass filter)	0.9609	0.9556	0.1998
FIR-ELM (low-pass filter)	0.9801	0.9889	0.1989

## Data Availability

The data used to support the findings of this study are available from the corresponding author upon request.
